The article "Sensory Processing and Autistic Traits: Mediation Effect of Frontal Alpha Asymmetry" was published in 2023. Journal: Occup Ther Int.

# Sensory Processing and Autistic Traits: Mediation Effect of Frontal Alpha Asymmetry

**DOI:** 10.1155/2023/5065120

**Published:** 2023-01-21

**Authors:** Deukgeun Yoon, Eun Young Kim

**Affiliations:** Department of Occupational Therapy, Soonchunhyang University, Asan-si 31538, Republic of Korea

## Abstract

A sensory processing approach can be used to intervene with behaviours in individuals with autistic symptoms. However, neural mechanisms linking sensory processing patterns and autistic features are less understood. The purpose of this study was to investigate whether frontal alpha asymmetry could mediate the relationship between atypical sensory processing and autistic traits. Seventy-three neurotypical young adults were included in this study. Resting-state brain activity was recorded using electroencephalography. After the recording, participants completed the Adolescent/Adult Sensory Profile and the Autism-Spectrum Quotient. Frontal alpha asymmetry was calculated by subtracting left frontal alpha power from right frontal alpha power. Correlation analysis was performed to find which sensory processing patterns were related to frontal alpha asymmetry and autistic traits. Mediation analysis was then conducted with sensory avoiding patterns as an independent variable, autistic traits as a dependent variable, and frontal alpha asymmetry as a mediator. Interrelations between higher sensation avoiding patterns, greater right-sided cortical activity, and increased autistic traits were found. The sensation avoiding patterns affected autistic traits directly and indirectly through right-sided cortical activity. Findings of the current study demonstrate a mediating role of frontal alpha asymmetry in the relationship between sensation avoiding patterns and autistic traits in neurotypical adults. This study suggests that sensation avoiding patterns and withdrawal-related emotions, which are associated with right-sided cortical activity, need to be considered to improve autism symptoms.

## 1. Introduction

Sensory processing can affect social interactions. Stimuli provided by others in a social context include various sensory elements such as voice, facial expression, and touch. How we process these sensory inputs is the basis of our social behaviours. Sensory processing difficulties are associated with social impairment [1, 2]. Atypical sensory processing is included in the diagnostic criteria for autism spectrum disorder (ASD) [3] characterized by deficits in social interaction and communication with restricted and repetitive behaviours. Since both sensory functioning and autistic traits exist along a spectrum, a relationship between sensory processing difficulties and autism symptomatology has been found not only in a clinical group with ASD [4] but also in the general population [5]. Individuals with sensory processing atypicalities are more likely to have social dysfunctions [6].

The article "Sensory Processing and Autistic Traits: Mediation Effect of Frontal Alpha Asymmetry" was published in 2023. Journal: Occup Ther Int.

To promote participation of individuals with autistic symptoms, sensory processing interventions may be applied by occupational therapy practitioners [7]. Evidence-based practices are supported by neuroscience research on sensory processing and autism [8]. However, to our knowledge, the neural mechanisms mediating the relationship between sensory processing patterns and autistic symptomatology have not been investigated yet. In the present study, we examined brain activity as a mediator between sensory processing patterns and autistic symptoms.

Frontal alpha asymmetry (FAA) is a neural mechanism involved in both sensory processing patterns and autistic traits [6]. FAA refers to a difference between right and left frontal alpha powers measured by electroencephalography (EEG) [9]. A positive value of FAA indicates that the right frontal alpha power is greater than the left frontal alpha power. Since frontal alpha has an inhibitory function [10], a positive FAA implies relative left-sided cortical activity. In contrast, a negative value of FAA indicates greater left frontal alpha power and relative right-sided cortical activity. The approach-withdrawal motivational model about FAA suggests that left cortical activity reflects approach properties whereas right cortical activity underpins withdrawal motivation [9, 11–13].

Sensory processing difficulties are linked to low FAA indicating relative right-sided cortical activity. Sensory hyporesponsiveness is associated with rightward cortical activity in young children having a sibling with ASD [14]. High sensory seeking patterns are related to rightward cortical activity and decreased social orienting [6]. FAA is also linked to ASD symptomatology [15]. The severity of ASD is associated with relative right-sided cortical activity [16]. In contrast, lower symptom levels of ASD are related to relative left-sided cortical activity [17]. Based on these previous findings, this study examined how sensory processing difficulties, FAA, and autistic symptoms are related to each other.

The relationship between atypical sensory processing and behaviours of individuals with ASD is mediated by anxiety [18], social orienting [6, 19], and emotion regulation [20]. A neural mechanism for these mediators has been suggested as FAA, an indicator of approach versus withdrawal motivation [9, 21–23]. These findings raise a possibility that FAA could mediate between atypical sensory processing and autistic traits. Thus, the objective of this study was to investigate the mediation effect of FAA on the association between sensory processing and autistic traits in neurotypical adults. To measure sensory processing, this study used the Adolescent/Adult Sensory Profile (AASP) on Dunn's model of sensory processing [24] because this model has been most commonly applied to measure sensory processing in autism [25]. In addition, the relationship between the AASP and autistic traits has been established in previous studies [26, 27]. This study hypothesized that high sensory processing atypicalities could predict high autistic traits through low FAA (relative right-sided cortical activity).

The article "Sensory Processing and Autistic Traits: Mediation Effect of Frontal Alpha Asymmetry" was published in 2023. Journal: Occup Ther Int.

## 2. Materials and Methods

### 2.1. Study Design

A cross-sectional design was used in this study, which was approved by the Institutional Review Board of Soonchunhyang University. Written consents were obtained from all participants. This research was conducted from August 2021 to October 2021.

### 2.2. Participants and Procedure

This study included 73 young adults (33 males and 40 females) with a mean age of 21.85 years (SD = 2.18). The sample size was determined based on previous studies examining FAA as a neural mediator between emotion and psychopathology [28–31]. Participants were recruited using a convenience sampling method at a university. Inclusion criteria were (1) typically developing individuals and (2) age of 18–28 years. Exclusion criteria were (1) coffee or tobacco consumption within 2 hours, (2) high impedance of electrodes, and (3) more than two standard deviations of FAA values. Participants received EEG recording before completing questionnaires to assess their sensory processing patterns and autistic traits. They were compensated with a gift corresponding to 3 USD for their participation time.

### 2.3. Measurements

#### 2.3.1. Electroencephalography Recording and Processing

To measure EEG, this study used the Cognionics Quick 20 dry EEG headset with 20 electrodes and a 500 Hz sampling rate. The EEG was recorded at 19 sites of 10-20 system electrode locations with reference to A1 (left ear). Electrooculography (EOG) and electrocardiography (ECG) were also measured to detect eye movements and heart artifacts using a CGX AIM physiological monitor. A resting-state eye-closed EEG recording was made in a quiet room. Participants were instructed to sit comfortably and close their eyes without moving during a 2-min recording.

EEG data were rereferenced with the Cz electrode [32] and band pass filtered from 0.5 to 30 Hz. Continuous EEG data were divided into 60 2-second epochs. Epochs containing noise and artifacts were excluded by visual inspection. An average of 48.86 epochs (SD = 8.75, range = 17 to 60) was analysed for each participant. Data of F3 and F4 were submitted for a fast Fourier transformation. The power spectral density of the alpha band (8–13 Hz) was averaged at each electrode. FAA was computed with the following formula: ln [right alpha(F4)] − ln[left alpha(F3)] [6]. A positive FAA means greater right frontal alpha power indicating relative left-sided cortical activity, whereas a negative FAA means greater left frontal alpha power indicating relative right-sided cortical activity. Analysis for the EEG data was performed using the EEGLAB v2021.1 [33] and MATLAB.

The article "Sensory Processing and Autistic Traits: Mediation Effect of Frontal Alpha Asymmetry" was published in 2023. Journal: Occup Ther Int.

#### 2.3.2. Adolescent/Adult Sensory Profile

The AASP is a self-report questionnaire on sensory processing patterns of daily life in individuals aged 11 years and over [24]. The AASP was designed on Dunn's model of sensory processing of neurological threshold (low versus high) and behavioural response (passive versus active), which provides quadrant score totals: low registration (high threshold and passive), sensation seeking (high threshold and active), sensory sensitivity (low threshold and passive), and sensation avoiding (low threshold and active). The AASP has six categories (taste/smell processing, movement processing, visual processing, touch processing, activity level, and auditory processing) and 60 items rated by a 5-point Likert scale (almost never, seldom, occasionally, frequently, and almost always), with a higher score indicating a higher frequency of the behaviour described in items. The current study used the Korean version of the AASP [34] with acceptable to good internal consistency.

#### 2.3.3. Autism-Spectrum Quotient

The Autism-Spectrum Quotient (AQ) is a self-report questionnaire on autistic traits in individuals aged 16 years and over [35]. The AQ has five subscales: social skill, attention switching, attention to detail, communication, and imagination. It includes 50 items rated by a 4-point Likert scale (definitely disagree, slightly disagree, slightly agree, and definitely agree), with a higher score indicating higher autistic traits. The current study used the Korean version of the AQ [36, 37] with acceptable to good internal consistency.

### 2.4. Data Analysis

Descriptive statistics were used for AASP quadrants (low registration, sensation seeking, sensory sensitivity, and sensation avoiding), FAA, and the AQ. Correlation analysis was performed between AASP quadrants, FAA, and the AQ. Sensory processing patterns that showed significant correlations with both FAA and the AQ were identified. Mediation analysis was then conducted with the sensory processing patterns as an independent variable, the AQ as a dependent variable, and the FAA as a mediator. This study used Baron and Kenny's approach to test the mediation model [38].

The article "Sensory Processing and Autistic Traits: Mediation Effect of Frontal Alpha Asymmetry" was published in 2023. Journal: Occup Ther Int.

## 3. Results

Table 1 shows the mean and standard deviation of AASP quadrants, FAA, and the AQ.

Sensation avoiding patterns of the AASP were significantly correlated with FAA and the AQ (Table 2). FAA and the AQ were also correlated with each other. Low registration patterns were correlated with the AQ, but not with FAA.

According to Baron and Kenny's procedure [38], the mediating effect was tested using three regression analyses. The first regression model showed that sensation avoiding patterns predicted FAA (*β* = −.25, *p* = .04), which explained 6% of the variance (*F* [1, 72] = 4.55, *p* = .04). The second regression model showed that sensation avoiding patterns predicted the AQ (*β* = .36, *p* = .002), which explained 12.6% of the variance (*F* [1, 72] = 10.28, *p* = .002). The third regression model showed that the AQ was predicted by both sensation avoiding patterns (*β* = .30, *p* = .01) and FAA (*β* = −.23, *p* = .05), which explained 17.4% of the variance (*F* [2, 72] = 7.40, *p* = .001). When FAA was included in the third regression model, the relationship between sensation avoiding patterns and the AQ was still statistically significant, although the significance was reduced. This result demonstrates that FAA is a partial mediator between sensation avoiding patterns and autistic traits (Figure 1).

## 4. Discussion

This study investigated the mediation effect of FAA on the relationship between sensory processing and autistic traits in neurotypical adults. Higher sensation avoiding patterns were related to increased autistic traits directly and indirectly through relative right-sided cortical activity. This result is consistent with previous findings showing that atypical sensory processing was associated with autistic traits [27] and right-sided cortical activity [6, 14]. This study further demonstrates that relative right-sided cortical activity partially mediates the contribution of sensation avoiding patterns to autistic traits.

In this study, sensation avoiding patterns among AASP quadrants showed significant correlations with both autistic traits and FAA. Compared to other quadrants, sensation avoiding patterns have been reported to have a stronger association with autism [26, 39, 40]. Sensation avoiding patterns are largely different between individuals with and without ASD [39, 40]. In addition, a relatively strong relationship between sensation avoiding patterns and overall autistic traits has been found in neurotypical adults [26]. These results support that sensation avoiding patterns are the most valid sensory characteristics for predicting autistic symptomatology.

The article "Sensory Processing and Autistic Traits: Mediation Effect of Frontal Alpha Asymmetry" was published in 2023. Journal: Occup Ther Int.

This study demonstrated that the relationship between sensation avoiding patterns and autistic traits was mediated by relative right-sided cortical activity of FAA. The rightward cortical activity is considered as a neural mechanism underlying withdrawal motivation [41] and its closely related emotion, anxiety [42, 43]. Anxiety, sensory processing abnormality, and autistic traits are interrelated in adults with or without ASD [27]. This interrelationship was also supported by the current study. This study further revealed how these components were related with each other by showing that the FAA, which is associated with anxiety, was a partial mediator for the relationship between sensation avoiding patterns and autistic traits.

Sensory processing patterns related to FAA differed between the current study and previous research. The relative right-sided cortical activity was associated with sensation avoiding patterns of neurotypical adults in the present study. However, it was associated with sensory hyporesponsiveness or sensory seeking patterns of infants having a sibling with ASD in previous studies [6, 14]. Such differences between the present study and previous studies might be attributed to developmental stages as the extent of sensory processing patterns changes with age [44, 45].

To establish neuroscientific evidence for sensory processing, event-related potential to stimuli has been examined for comparisons between typically developing children and children with sensory processing disorder [46–49]. Children with sensory processing disorder showed deviant brain activity that indicates inefficient sensory function. A recent study has applied resting-state EEG to investigate sensory processing disorder [50]. It was found that individuals with sensory overresponsiveness exhibited reduced alpha power reflecting alert and vigilance states, suggesting that this resting-state activity could mediate between sensory overresponsiveness and pain response. Aligned with these findings, the current study provides additional neurophysiological evidence for sensory processing.

This study has implications for occupational therapy practice. Sensation avoiding patterns and rightward cortical activity contributed to autistic traits, suggesting that occupational therapy practitioners need to consider avoidance from sensory input and withdrawal-related emotion when dealing with autistic symptomatology such as social and communication difficulties. The mediation model of sensation avoiding, FAA, and autistic traits raises a possibility that the intervention for sensory processing may attenuate autistic behaviours directly and indirectly by modulating brain activity. Improvement of sensory processing may shift frontal activity from the right cortex associated with withdrawal motivation to the left cortex related to approach motivation, which in turn may reduce autistic symptoms. This study provides evidence of the neural mechanism linking sensory processing and autistic features in occupational therapy practice.

The article "Sensory Processing and Autistic Traits: Mediation Effect of Frontal Alpha Asymmetry" was published in 2023. Journal: Occup Ther Int.

Ayres Sensory Integration® (ASI) [51] is an evidence-based practice for individuals with autism [52] that aims to improve sensory processing skills with sensory activities that can promote sensory awareness, affect and arousal regulation, and motor control. The ASI is provided as a tailored intervention considering clients' abilities, choices, and intrinsic motivations, enabling clients to give adaptive responses in a positive atmosphere [53]. These ASI elements may facilitate approach motivation related to leftward cortical activity. The present study demonstrates that FAA is a possible neural mechanism between ASI and the improvement of autistic features.

FAA shows more leftward cortical activity after meditating or mindfulness-based stress reduction training [54, 55], indicating that these interventions can increase positive emotion and approach motivation. Mindfulness is defined as intentional attention and awareness to the present moment without judging and reacting to it, which contains sensory processing components such as noticing and accepting sensations [56, 57]. High sensory processing sensitivity characterized by low sensory threshold and being easily stimulated [58] is associated with low mindfulness, which in turn is related to psychological problems [59]. It has been proposed that mindfulness training including awareness and acceptance of sensations may improve psychological health for highly sensitive people [59, 60]. Current findings and previous findings imply that mindfulness training as well as a sensory integration approach may promote appropriate sensory processing, which might be reflected in more leftward cortical activity, consequently reducing autism symptoms.

This study has some limitations. First, the current study was focused on neurotypical adults, considering that the relationship between sensory function and autistic traits was similar between individuals with and without ASD [26]. However, to expand this study into clinical settings, future studies should include participants with ASD. Second, caution is needed when generalizing these results to children since sensory processing changes with age [61]. A further study is needed to investigate age-related changes in the relationship of sensory processing with neural activity and autism symptoms. Third, we did not ask participants about their use of medication. Given that FAA is not altered by medication [62], it is unlikely that medication has affected our EEG results. However, to rule out the effect of medication completely, it is necessary to check medication in further studies. Fourth, although the AASP can assess sensory processing patterns in daily life, it depends on subjective self-report. Sensory processing can be objectively measured with physiological reactivity to sensory stimuli [63]. Further studies are needed to investigate relationships between sensory reactivity, FAA, and autistic traits.

The article "Sensory Processing and Autistic Traits: Mediation Effect of Frontal Alpha Asymmetry" was published in 2023. Journal: Occup Ther Int.

## 5. Conclusions

This study demonstrates that FAA partially mediates the relationship between sensory processing and autistic traits in neurotypical adults. Sensation avoiding patterns influenced autistic traits directly and indirectly through relative right-sided cortical activity. This study suggests sensation avoiding patterns and withdrawal motivation as potential important intervention targets for people with autistic traits. The present study can deepen our understanding of neurophysiological mechanisms mediating between sensory processing and autistic traits.

## Figures and Tables

**Figure 1:** Direct effect of sensation avoiding patterns on autistic traits and indirect effect via frontal alpha asymmetry. Note: ^∗^*p* < .05 and ^∗∗^*p* < .01.

**Table 1:** Descriptive statistics of measurements.

Measurements	Mean (SD)
AASP	
Low registration	28.68 (7.45)
Sensation seeking	38.97 (7.15)
Sensory sensitivity	36.38 (9.28)
Sensation avoiding	37.30 (7.07)
FAA	0.02 (0.06)
AQ	17.89 (5.44)

Note: AASP: Adolescent/Adult Sensory Profile; FAA: frontal alpha asymmetry; AQ: Autism-Spectrum Quotient; SD: standard deviation.

**Table 2:** Correlations between AASP quadrants, FAA, and the AQ.

	AASP									
	Low registration		Sensation seeking		Sensory sensitivity		Sensation avoiding		AQ	
	*r*	*p*	*r*	*p*	*r*	*p*	*r*	*p*	*r*	*p*
FAA	−.19	.10	07	.54	−.08	.53	−.25^∗^	.04	−.30^∗∗^	.01
AQ	.27^∗^	.02	−.17	.15	.05	.70	.36^∗∗^	.002	1	

Note: ^∗^*p* < .05 and ^∗∗^*p* < .01. AASP: Adolescent/Adult Sensory Profile; FAA: frontal alpha asymmetry; AQ: Autism-Spectrum Quotient.

## Data Availability

The data used to support the findings of this study are available from the corresponding author upon request.
